# Word Sequential Using Deep LSTM and Matrix Factorization to Handle Rating Sparse Data for E-Commerce Recommender System

**DOI:** 10.1155/2021/8751173

**Published:** 2021-12-07

**Authors:** Hanafi, Burhanuddin Mohd Aboobaider

**Affiliations:** ^1^Faculty of Computer Science, University of Amikom Yogyakarta, Yogyakarta 55283, Indonesia; ^2^Faculty of Information and Communication Technology, Technical University of Malacca, Malacca 76100, Malaysia

## Abstract

Recommender systems are essential engines to deliver product recommendations for e-commerce businesses. Successful adoption of recommender systems could significantly influence the growth of marketing targets. Collaborative filtering is a type of recommender system model that uses customers' activities in the past, such as ratings. Unfortunately, the number of ratings collected from customers is sparse, amounting to less than 4%. The latent factor model is a kind of collaborative filtering that involves matrix factorization to generate rating predictions. However, using only matrix factorization would result in an inaccurate recommendation. Several models include product review documents to increase the effectiveness of their rating prediction. Most of them use methods such as TF-IDF and LDA to interpret product review documents. However, traditional models such as LDA and TF-IDF face some shortcomings, in that they show a less contextual understanding of the document. This research integrated matrix factorization and novel models to interpret and understand product review documents using LSTM and word embedding. According to the experiment report, this model significantly outperformed the traditional latent factor model by more than 16% on an average and achieved 1% on an average based on RMSE evaluation metrics, compared to the previous best performance. Contextual insight of the product review document is an important aspect to improve performance in a sparse rating matrix. In the future work, generating contextual insight using bidirectional word sequential is required to increase the performance of e-commerce recommender systems with sparse data issues.

## 1. Introduction

The development of recommender systems (RS) aims to support marketing by increasing target selling. RS has been developed to generate product recommendations to help customers choose a product automatically. RS has been adopted in many large e-commerce companies such as Amazon, Google, Netflix, iTunes, Facebook, eBay, and Alibaba. Many experts explained that the successful adoption of recommender systems could significantly influence the marketing target [1]. Most e-commerce companies in the world decided to implement recommender systems to increase service satisfaction for their company by making it more enjoyable for the customers to look for the products they need. A recommender system is an essential tool to promote the products and services for many online websites and mobile applications. For instance, 80% of the movies watched on Netflix came from recommendations [2], and 60% of video clicks on YouTube came from home page recommendations [3]. According to Schafer et al. [4], sales agents with recommendations from the NetPerceptions system achieved a 60% higher average cross-sell value and 50% higher cross-sell success rate than agents using traditional cross-sell techniques, based on experiments conducted at a UK-based retail and business group.

Based on a general algorithm approach [5–9], e-commerce RS are divided into four types: (1) content-based, which is a method to generate recommendations according to a product classification approach—it involves information retrieval to generate product recommendations; (2) knowledge-based, which develops a specific and/or necessary recommendation and includes providing product information rarely needed for individual purposes (e.g., houses, loans, insurance, and cars.); (3) demographic-based, which refers to product recommendations established according to demographic information; and (4) collaborative filtering, which is a mechanism used to produce recommendations based on the user's behaviour in the past, such as a product rating, product review, comment, testimony, and purchase.

Collaborative filtering is considered as the most successful recommendation technique to be implemented in many large e-commerce companies, as it can provide recommendations with special character information such as providing product fit information, giving relevant information, having highly accurate recommendations, and being serendipitous [10]. In common use, most collaborative filtering adopts ratings as explicit feedback for the basic calculation method to compute the similarity in users' behaviors. Unfortunately, the number of ratings is very small. In general, customers are lazy to give ratings for a product. GroupLens product is the most popular e-commerce dataset containing the movie rating matrix, which includes ML-100k, ML-1M, ML-10M, and ML-20M [11]. Amazon is the second most popular dataset that contains ratings of only less than 1%. The most common problem in collaborative filtering is generating rating prediction in sparse data rating matrix conditions. Traditional collaborative filtering implemented memory-based popular neighborhood model to obtain rating prediction. Most traditional statistical approaches have been created by several researchers during the early emergence of collaborative filtering in the mid-90s. Collaborative filtering calculates the nearest neighbor among users with similar behaviors with respect to product interest. Unfortunately, the findings for the calculation of a neighbor's vector require heavy computation in large-scale datasets. From a practical point of view, memory-based methods adopt neighbor heuristics, so they may meet several challenges on large datasets. The neighborhood algorithm uses several kinds of traditional statistic mechanisms, such as cosine similarity, Spearman's rank, Pearson's correlation, etc. An example of the nearest neighborhood model to calculate the similarity in user behaviors is shown in the following equation:

(1) $$\begin{array}{c} \text{sim}\left(u,v\right)=\frac{\sum_{v\in N_{i}\left(u\right)}\text{sim}\left(u,v\right)\left(r_{vi}-{\hat{r}}_{v}\right)}{\sum_{v\in N_{i}\left(u\right)}\text{sim}\left(u,v\right)}. \end{array}$$

The memory-based model results in a simpler product recommendation, which is easy to be implemented and requires no training data to gain product ranking. This is the benefit of memory-based collaborative filtering. However, memory-based face a serious problem with respect to scalability. The increasing number of users and products may cause computation levels to be heavy or high. This is the essential reason that emerges in the modern collaborative filtering model, popularly known as a model-based or latent factor model that functions to exploit the latent correspondents between the user and product relationship.

Matrix factorization, popularly called model-based, becomes more popular over memory-based since the Netflix competition has been held in 2006. Model-based involves matrix factorization to handle the completion of the rating matrix. In fact, the matrix factorization model was introduced by Sarwar et al. [12] in the early 2000s by using a low-rank dimensional implementation called Singular Value Decomposition (SVD). SVD tried to calculate the latent relationship between the user and items. Koren et al. [13] proposed a novel SVD to improve the traditional SVD in order to increase its effectiveness in generating rating prediction, including time-stamp rating given by the user that named temporal effects, namely, TimeSVD. According to an experiment report, TimeSVD succeeded in improving the performance of Sarwar et al.'s traditional SVD. Koren et al. attempt to enhance the previous work using SVD combined with neighborhood representation [14]. Another model considers mathematical and statistical approaches that only consider the rating information proposed by Salakhutdinov and Mnih [15]. Salakhutdinov and Mnih popularized the probabilistic approach to be integrated with matrix factorization, called probabilistic matrix factorization (PMF). The PMF model is claimed to be an extended version of the SVD model. PMF works by transforming user and item information into a 2D vector dimension using Gaussian normal distribution. The PMF model succeeds in generating rating prediction in large datasets, and, surprisingly, it is also robust when faced with imbalanced data.  Figure 1 shows an example of the rating matrix representation of collaborative filtering, where the red color represents the unrated items.

The latent factor models have succeeded in increasing the performance of an accurate rating prediction based on memory. However, there was a shortcoming when dealing with extremely sparse data conditions. Several experts have proposed various models to support latent factor performance. The researcher considered integrating the product review with matrix factorization. One of the researchers is Ling et al. [16], who proposed a novel model using item review to support the latent factor model. A document of a product review is the representation of a user's satisfaction over a product. In that research, Ling et al. used the Latent Dirichlet Allocation (LDA) model to interpret product review documents. The LDA model proposed by Ling et al. succeeded in refining the traditional latent factor using SVD, TimeSVD, and PMF. Another model suggested by Wang and Blei [17] also proposed a model using LDA to interpret product documents and integrate them with a latent factor called Collaborative Topic Regression (CTR). Wang and Blei employed probabilistic matrix factorization to produce rating prediction. Both LDA models that were integrated into matrix factorization were successful in increasing the effectiveness in generating rating prediction.  Table 1 shows the previous state-of-the-art methods, including the traditional latent factor and the hybrid between the latent factor and product review document.

The interpretation of text documents becomes an essential factor in the field of Natural Language Processing (NLP). The traditional Bag of Words (BOW) mechanism was a popular method in the early decades and has been applied in several commonly used applications in the field of NLP. Unfortunately, the LDA model fails to capture the contextual understanding of sentence documents. Some experts have tried to refine the BOW mechanism by exploiting deep learning models. For example, for sentence classification, they applied the Convolutional Neural Network (CNN) that has been successful in refining accuracy levels in the traditional sentence classification in previous works [23]. According to current studies, in recent years, the application of CNN in recommender system territory has been proposed by Kim et al. [20]. Another researcher applied a subclass of deep learning, called autoencoder (AE), which aims to refine the performance of matrix factorization [24]. According to an experiment report, using a deep learning class, either AE or CNN, is successful in increasing the effectiveness of rating prediction as compared to the traditional BOW mechanism. However, according to contextual semantic insight perspective, most of the models ignored the contextual understanding of product documents. The contextual understanding of a sentence can be captured by the following two essential aspects explained as follows: (1) considering word order or word sequence and (2) considering subtle words to each other.

A novel collaborative filtering method involving social information representation, called SSDAE, integrates collaborative filtering based on PMF and the social behaviour of the user [25]. The different way of this approach is that it involves social information documents to support matrix factorization as a latent factor representation approach. Several previous works only adopted product document representation, which may have had the limitation of user information representation. Similar to ConvMF, SSDAE can also consider PMF as a latent factor machine in order to obtain rating prediction.

Long Short-Term Memory (LSTM) is a subclass of deep learning. LSTM has a unique characteristic over other deep neural networks in which it can recognize sequential information aspects. This is an important aspect of learning contextual semantic understanding in the context of a document. LSTM can be integrated into a recommender system algorithm to improve sentence document interpretation. The implementation of LSTM is expected to support matrix factorization to increase the effectiveness in the generation of rating prediction. In this research, we proposed a novel method by including LSTM to transform the product review document into a 2D semantic latent space and integrate it with probabilistic matrix factorization (PMF). We evaluated our model using the evaluation metrics based on Root Mean Square Error (RMSE). We also applied our model to two real datasets: MovieLens (ML-1M) and Amazon Information Video (AIV). Our novel algorithm model includes LSTM-GLOVE-PMF. This research contribution is presented in Table 2, where contextual understanding using word embedding and LSTM is a novel hybrid latent factor model. Our proposed model is called LSTM-PMF.

In this paper, we demonstrated two contributions, including (a) a novel model to capture the contextual documents by considering the sequential aspects of LTSM and word embedding and (b) integration of the contextual documents into probabilistic matrix factorization. Thus, this experiment results require evaluating the aims to identify the performance achievement using RMSE evaluation metrics.

## 2. Materials and Methods

This research exploited two essential methods, namely, PMF and LSTM. PMF is responsible for generating rating predictions by learning the correspondence between items and user's information. Meanwhile, the role of LSTM is to support latent factors in generating rating prediction to enhance its effectiveness. LSTM works by utilizing product review documents to gain a 2D space document vector. The details of our proposed method involve two essential mechanisms that are explained in the three sections below.

The architecture of LSTM-PMF is presented in Figure 2. The architecture figure consists of five-layer stages. Every layer territory carries out a specific task. The first layer on the top is responsible for collecting datasets, including ML-1M, ML-10M, and AIV. The second layer is to conduct preprocessing using an NLTK module and to develop the preprocessing results using word embedding based on GLOVE. After being processed in the second layer, the third layer territory will generate contextual understanding with the word sequential detection process using LSTM. This process is also responsible for transforming the document product review into a 2D vector space 50. The fourth layer is responsible for bridging the user latent space and item document latent space. The second task of this layer is to generate a rating prediction by learning the correspondence between variable *U* as a user representation and vector *V* as an item representation. In this layer, the probabilistic matrix factorization links the item document and user representation. The last layer is responsible for evaluating the rating prediction output using RMSE evaluation matrices that include several standards. A detailed description of the computation method is presented in the methodology section.

The Materials and Methods section contains sufficient detail so that all procedures can be repeated. It may be divided into headed sections in case several methods are described.

### 2.1. Probabilistic Matrix Factorization

Since the latent factor model has been exploited in collaborative filtering in early 2006, several researchers have tried to solve the major problems, specifically regarding the sparse data issue. The latent factor model based on matrix factorization is a very effective method to generate rating prediction. Rating is an essential factor in producing product recommendations. Using a rating matrix obtained from customers, the recommender machine produces a product ranking, which is then presented to the customer or customer candidate. The basic principle of matrix factorization is to rotate, invert, and reduce the matrix content. Therefore, a complete rating matrix can then be obtained [27]. SVD is an example of a successful matrix factorization model with a low-rank dimensional that is used to learn the correspondence between the item and users. PMF is claimed to be an extension of SVD that considers the Gaussian normal distribution to generate a rating distribution based on the probabilistic work mechanism rule. An illustration of the essential factorization model of the rating matrix for two lower-dimensional matrices can be depicted as follows: for example, *M* represents the movie, *N* represents the users, and an integer represents the rating value starting from *1* to *K*. *R*_*ij*_ is the representation of user *i* with movie *j.* Also, *U* ∈ *R*^*D*×*N*^, *V* ∈ *R*^*D*×*M*^. The variables of *U* and *V* become the representation of the latent user and movie matrices, respectively. The rating prediction obtained by a given user *i* for movie *j* can be computed as *R*_*ij*_=*U*_*i*_^*T*^, *V*_*j*_. The illustration for the basic concept of matrix factorization based on collaborative filtering can be presented in Figure 3.

The idea of PMF was initially proposed by Salakhutdinov and Mnih when the Netflix competition was held in mid-2006 [15]. PMF successfully refined Netflix's recommender system up to 4%. Unfortunately, with less than 10% achievement, the PMF model could not win the competition. PMF's categorical probabilistic linear approach used the Gaussian normal distribution and the vector representation of a user and movies acquired from the distribution of a rating correspondents. A detailed formulation of the distribution is given the following equation:

(2) $$\begin{array}{c} p\left(R_{ij}|U_{i},V_{j},\sigma^{2}\right)=Ν\left(R_{ij}|U_{i}^{T}V_{j},\sigma^{2}\right). \end{array}$$

Aimed at transforming into a latent feature vector of the item, this model considers using a zero-mean spherical Gaussian prior to a detailed equation as follows:

(3) $$\begin{array}{c} p\left(V|\sigma_{V}^{2}\right)=\prod_{j=1}^{M}N\left(V_{i}|0,\sigma_{V}^{2}I\right). \end{array}$$

Aimed at transforming into a latent feature vector of the user, this model considers using a zero-mean spherical Gaussian prior to a detailed equation as follows:

(4) $$\begin{array}{c} p\left(U|\sigma_{U}^{2}\right)=\prod_{i=1}^{N}N\left(U_{i}|0,\sigma_{U}^{2}I\right). \end{array}$$

### 2.2. Capturing the Contextual Insight of a Product Document Using LSTM

The contextual understanding of a sentence can be understood by considering its word sequence and subtly words. Most neural network technologies generalize a process from the input to produce an output. Unlike most neural network models, LSTM pays attention to the process of input by observing the sequence of processes with time series in the input process. One interesting aspect of the LSTM method is the notion where it is possible to link past information stages and the current process, for instance, enabling past video frames to introduce an understanding to the current video. Referring to the context of natural language, it is essential to reveal the contextual understanding of a sentence document, where the sequential perspective is an essential aspect to be explored; this is due to the semantic insight point of view. A specific type of RNN is Long Short-Term Memory that is commonly known as LSTM. It is specially performed for long dependency learning. The LSTM is also an enhancement of the RNN architecture. It was first published by Hochreiter and Schmidhuber [28]. The model has been improved and popularized by many people for being suitable for several tasks in the field of computer science. Some formulas explain how the hidden state of LSTM can be used to learn sequential aspects from an input. The workings of the hidden state of LSTM are explained in Figure 4 and equation (5).

The hidden layer of LSTM consists of several processes to accommodate the input layer, output layer, the previous process of the hidden state, and the output of the hidden state. The ability of LSTM to detect sequential aspects leads to several essential computation processes in the hidden state. A detailed explanation of LSTM's work is shown in equation (5). Every variable obtains an output due to the learning process based on some calculations that involve several aspects, as follows:

(5) $$\begin{array}{c} i=\sigma \left(x_{i}U^{i}+S_{t-1}W^{i}\right),\\ f=\sigma \left(x_{i}U^{f}+S_{t-1}W^{f}\right),\\ o=\sigma \left(x_{t}U^{o}+S_{t-1}W^{o}\right),\\ g=\tanh\left(x_{i}U^{g}+S_{t-1}W^{g}\right),\\ c_{t}=c_{t}-Of+gOi,\\ h_{t}=\tanh\left(c_{t}\right)-O_{o}gOi. \end{array}$$

 
*i*, *f*, *o*: *i* represents input, *f* represents forget, and *o* represents output gates. All of them own similar equations and have only different parameter matrices. These are known as gates due to the sigmoid rule that determines the value as either 0 or 1.
 
*g*: It represents the hidden state, which is calculated based on the existing input and the past hidden state.
 
*c*_*t*_: It represents the internal memory of the hidden state. It is a combination of the previous memory *c*_*t*−1_ that is multiplied by a forget gate and the new hidden state *g* that is multiplied by the input gate.
 
*h*_*t*_: It represents the memory of the hidden state. The computed output of the hidden state on *h*_*t*_ is multiplied by the output gate.

### 2.3. Preprocessing of Product Review Document

In this research, preprocessing is carried out as a standard research process to extract the raw documents based on some previous work standards [24, 29]. Preprocessing is necessary for the computational process to produce a document with representative meaning. A detailed description of the preprocessing step is given in Table 3 below.

### 2.4. Transform the Raw Document into 2D Vector Space

After going through some of the preprocessing phases presented above, the results are transformed into a 2D vector space. In this process, the contextual meaning is expected to be successfully captured so that the user's expression can be correctly understood, such as understanding the meaning of the user's expression. The explanation of several processes in transforming the product review document into a 2D vector space is presented in Figure 5. In the beginning, datasets from AIV were collected. The product review documents selected were only those related to the MovieLens movie catalog. According to the LSTM mechanism, every word vector is like the output from word embedding obtained from the GLOVE processing, placed in a unique hidden layer [30]. As a result of the previous section, every product owns a product review containing 300 words in the form of word vector representation. The complete process for transforming the raw document into 2D vector 50 is explained in Figure 5.

After the product review of the document training set process using LTSM and word embedding is finished, the output in the form of 2D vector 50 would be integrated into probabilistic matrix factorization, which was expected to support handling sparse data problems powerfully. PMF plays an important role in bridging the user latent model and item document latent model in order to learn the correspondence between them.

### 2.5. Hybrid LSTM and PMF

According to the LSTM point of view, it is not appropriate to use regression applications such as rating prediction in a collaborative filtering recommender system. The output of LSTM in the form of a 2D vector representation cannot be directly applied to predict the rating. Aimed at handling the above problem, LSTM needs to be integrated with matrix factorization, such as PMF. PMF is responsible for calculating the relationship between the latent model of users and the product latent space that strengthens the user and item correlation. For example, we have *N* as the representation of the user and *M* as the representation of the item. The formula to calculate the rating value is *R* ∈ ℝ^*N*×*M*^ matrix, while the formula for user representation and item representation is given by *U* ∈ ℝ^*K*×*N*^ and *V* ∈ ℝ^*K*×*N*^, respectively. Finally, the table of products is obtained by *U*^*T*^*V*, with the objective to recalculate the table rating matrix *R*. Following the role of the probabilistic perspective, the normal distribution representation is as follows:

(6) $$\begin{array}{c} p\left(R|U,V,\sigma^{2}\right)=\prod_{i=1}^{N}\overset{M}{\underset{j-1}{\prod }}{\left[N\left(R_{ij}|U_{i}^{T}V_{j},\sigma^{2}\right)\right]}^{I_{ij}}, \end{array}$$

where *µ* is the mean of population number, *σ*^2^ is variance value, and*i*_*j*_ is an indicator function as a generative model for user latent models.

The probabilistic model is a key factor in developing the LSTM-PMF model.  Figure 6, as presented below, shows the role of PMF to bridge the item latent representation and user latent model within a document vector representation. The blue color is a matrix factorization territory consisting of *U*, *V*, and *R*. The red color is the item document representation territory. GLOVE-LSTM supports document representation to generate the weight of *W* variables.

The LSTM-PMF model, as illustrated above, obtained both item and user latent model processes. A detailed explanation of the two processes has been given in the following sections.

### 2.6. User Latent Model Representation

User information representation collected by MovieLens contains user and rating information only. The user latent model territory uses zero mean spherical Gaussian prior by involving the variance value of user data *σ*^*2*^, and the following equation is given:

(7) $$\begin{array}{c} p\left(U|\sigma_{U}^{2}\right)=\prod_{i-1}^{N}N\left(U_{i}|0,\sigma_{U}^{2}I\right). \end{array}$$

### 2.7. Item/Product Latent Model Representation

Item information representation is collected from AIV in the form of item documents. A 2D vector 50 is obtained after passing several processes following the LSTM mechanism. According to the probabilistic point of view, the item latent model follows the following equation:

(8) $$\begin{array}{c} p\left(\left(V|W,X,\sigma_{W}^{2}\right.\right.=\prod_{j}^{M}N\left(v_{j}|\text{lstm}\left(W,X_{j}\right)\sigma_{W}^{2}I\right). \end{array}$$

Meanwhile, the item variable *v*_*j*_ is obtained as follows:

(9) $$\begin{array}{c} v_{j}=\text{lstm}\left(W,X_{j}\right)+\varepsilon_{j}. \end{array}$$

The probability density function in the probabilistic point of view with normal distribution can be obtained as follows:

(10) $$\begin{array}{c} \varepsilon_{j}∼N\left(0,\sigma_{V}^{2}I\right). \end{array}$$

Document latent representation produced by word embedding and LSTM is required to be transformed to normal distribution and follows the following equation:

(11) $$\begin{array}{c} p\left(W|\sigma_{W}^{2}\right)=\prod_{k}N\left(W_{k}|0,\sigma_{W}^{2}\right). \end{array}$$

Optimization of the learning latent space model between variables *U*, *V*, and *W* is explained in the following sections below.

### 2.8. Optimizing the Latent Space Dimension and Generating the Rating Model

The optimization process works to strengthen the correspondence between the overall variables such as user latent variable, item latent variable, share weight variable, and bias variable of LSTM. We adopted the model to apply Maximum A Posteriori (MAP) [15]. MAP is a Bayesian statistic aimed to calculate an unknown quantity. It is similar to the posterior distribution. Specifically, it aims to optimize the learning variable in consideration of the MAP application. This method adopted log a posteriori through user and movie features using hyperparameters. The complete formula of MAP is presented as as follows:

(12) $$\begin{array}{c} \underset{U,V,W}{\max}p\left(U,V,W|R,X,\sigma^{2},\sigma_{U}^{2},\sigma_{v}^{2},\sigma_{W}^{2}\right)=\;\underset{U,V,W}{\max}\left[p\left(R|U,V,\sigma^{2}\right)p\left(U|\sigma_{U}^{2}\right)p\left(V|W,X,\sigma_{V}^{2}\right)p\left(W|\sigma_{W}^{2}\right)\right]. \end{array}$$

This experiment also applied a negative logarithm to learn the user and item feature for the training process with minimized loss function ℒas follows:

(13) $$\begin{array}{c} ℒ\left(U,V,W\right)=\sum_{i}^{N}\sum_{j}^{M}\frac{I_{ij}}{2}{\left(r_{ij}-u_{i}^{T}v_{j}\right)}_{2}+\frac{\lambda U}{2}u_{i2}+\frac{\lambda V}{2}\overset{M}{\underset{j}{\sum }}v_{j}-\text{lstm}{\left(W,X_{j}\right)}_{2}+\frac{\lambda W}{2}\overset{W_{k}}{\underset{k}{\sum }}W_{k2}. \end{array}$$

where *λ*_*U*_ is *σ*^2^/*σ*_*U*_^2^ as the representation of users' variance, *λ*_*v*_ is *σ*^2^/*σ*_*V*_^2^ as the representation of item variance, and *λ*_*W*_ is *σ*^2^/*σ*_*W*_^2^ as the representation of *W* variance.

Thus, to develop a coordinate descent, the researchers used the squared function to learn the correspondent *U*, *V*, and *W*. The following equation represents the coordinate descent and is given as follows:

(14) $$\begin{array}{c} U_{i}⟵{\left({\text{VI}}_{i}V^{T}+\lambda_{U}I_{K}\right)}^{-1}{\text{VR}}_{i}\text{ and }V_{j}⟵{\left({\text{UI}}_{j}U^{T}+\lambda_{V}I_{K}\right)}^{-1}\left({\text{UR}}_{j}+\lambda_{V}\text{lstm}\left(W,X_{j}\right)\right). \end{array}$$

We used a backpropagation algorithm to optimize *W*, in which *W* represents the weight variable and bias variable for every layer, which is an important step in it. Aimed at optimizing every layer, including *V*, *U*, and *W*, the update mechanism until convergence is required. The formula used to predict the unknown rating is given below:

(15) $$\begin{array}{c} r_{ij}\approx E\left[r_{ij}|u_{i}^{T}v_{j},\sigma^{2}\right]=u_{i}^{T}v_{j}=u_{i}^{T}\left(\text{lstm}\left(W,X_{j}+\varepsilon_{j}\right.\right). \end{array}$$

### 2.9. Datasets

MovieLens is one of the most popular datasets to conduct an e-commerce experiment. It was initially developed in 1997 by the School of Computing, University of Minnesota [11]. Majority recommender system experiments applied MovieLens datasets [11, 31]. It aimed to obtain information for personal suggestions. MovieLens datasets contain some categories that depend on the number of ratings, number of users, number of products, and the density level of sparse ratings. This experiment adopted the product review document from AIV, which is a popular dataset collected from Amazon [32–34]. The description of the dataset's characteristics is presented in Table 4.

This experiment involves 2 MovieLens categories, including ML-1M that contains 1 million ratings with a sparse level of 4.64% and ML-10M that contains 10 million ratings with a sparse level of 1.41%. This is an important factor to be observed in the performance of LSTM-PMF in various sparsity level conditions.

### 2.10. Evaluation Result

The performance of LSTM-PMF needs to be evaluated. RMSE evaluation matrices are the most popular method to evaluate the effectiveness of rating predictions [35, 36]. The scenario of the experiment is divided into nine parts, in which every part splits the dataset by 10 percent interval ratio, including 10 : 90, 20 : 80, 30 : 70, 40 : 60, 50 : 50, 60 : 40, 70 : 30, 80 : 20, and 90 : 10.

The output of the training process was evaluated using the RMSE evaluation matrix. The formula of the evaluation matrices is given by the following equation:

(16) $$\begin{array}{c} \text{RMSE}=\sqrt{\frac{\sum_{i,j}^{N,M}{\left(r_{ij}-{\hat{r}}_{ij}\right)}^{2}}{\left(\text{total}\#\text{rating}\right)}}. \end{array}$$

In essence, the result of rating prediction obtained by LSTM-PMF is compared with the actual rating based on dataset resources.

### 2.11. Experiment Tools

In this research, some tools and library modules were used to make sure the experiment follows the standards of previous work, including deep learning tools, hardware, and supporting modules. The listing of tools and libraries are presented in Table 5.

## 3. Results and Discussion

The results of the rating prediction using several training data scenarios are demonstrated in the following figures. The results and comparisons consider presenting the existing state of the art using traditional matrix factorization based on PMF and the previous best result based on CNN and matrix factorization. This experiment consisted of 2 training scenarios, including implementation on real datasets from ML-1M and ML-10M.

### 3.1. Experiment Scenario on ML-1M

Dataset ML-1M was categorized into the middle dataset from the scalability point of view and a normal sparse level, with a density factor of 4.64%. Aimed at investigating the performance of our model, we implemented the model into real datasets. The MovieLens dataset represents rating sparse data without product review. Meanwhile, Amazon is a categorized e-commerce dataset without a rating matrix, with rich product information in terms of product review document. The nine scenarios of the training evaluation process are demonstrated in Figures 7to 15. The experiment was applied to ML-1M and Amazon datasets with per 10% interval sparseness levels. The training process included the PMF, CNN-PMF, and LSTM-PMF models, respectively. The complete training process and RMSE evaluation results are shown in the nine figures below.

According to the experimental results as depicted in the nine figures above, the use of product reviews is very helpful in enhancing the effectiveness of rating predictions even in extremely sparse rating conditions. As reported in Figure 15, it can be inferred from the model to apply PMF where this model does not apply product reviews, while CNN-PMF and LSTM-PMF involve product review documents obtained outperform in accuracy and are faster to achieve convergence. Moreover, the implementation of the LSTM model aimed at capturing the contextual meaning of the product reviews achieves outperformance over the CNN model due to the fact that the LSTM model produces a higher share weight over CNN.

As shown in Figure 16, the model applying product review documents is superior in comparison to the traditional PMF model even in the extremely sparse rating condition (e.g., 10%, 20%, 30%, and 40%). The implemented LSTM model slightly outperforms in each training scenario over CNN. As reported in Table 6, it is believed that LSTM is successful in improving the traditional latent factor using PMF and modern deep learning using CNN. LSTM-PMF improved 15% on an average as compared to the traditional PMF model and improved by 0.71% on an average as compared to CNN-PMF.

### 3.2. Experiment Scenario on ML-1OM

The dataset ML-10M was categorized as a large dataset from a scalability point of view. This category was quite extreme in its sparsity level, in which the density factor was 1.4%.

The training result, as shown in Figures 17to 25, showed that LSTM-PMF outperformed the traditional matrix factorization significantly; however, it lost CNN-PMF.

A summary of the evaluation training scenarios on ML-10M is shown in Figure 26. LSTM-PMF significantly succeeded in improving the effectiveness of the rating predictions as compared to PMF. However, the rating number was very sparse, with a density level of 1.4%.

A detailed comparison of ML-10M is presented in Table 7. It can be concluded that LSTM was successful in refining the effectiveness of the rating prediction, either in traditional or modern matrix factorization, by incorporating the deep learning classes based on CNN. LSTM-PMF achieved 10% on an average over the traditional PMF and performed 1.41% on an average over CNN-PMF. In this case, LSTM-PMF was more powerful and achieved significant performance in normal conditions over sparse rating levels such as 10/90 and 20/80, in which the performance achieved was similar to that of CNN-PMF. The achievement was quite significant when this model was applied to the 50 : 50 training ratio above. Compared to the ML-1M results, the performance of LSTM-PMF was more powerful, with a significant performance of 1.44% on average achieved over that of CNN-LSTM.

The significant performance of LSTM-PMF over the traditional PMF was due to the document latent vector, which is a key factor for better achievement. Latent factor vector document representation in *W* supports the item latent model *V* to learn the correspondence between the item and users. The implementation of document latent representation also increased effects in the effectiveness of the training process, in which a smaller number of iterations are required to achieve convergence over the traditional PMF.

According to the ML-1M experiment report, document vector representation also supported the item latent vector to increase the performance to more than 15% on an average over PMF. In the larger datasets of ML-10M, this model consistently outperformed PMF on every training set scenario, reaching up to 10% on average over PMF. Moreover, LSTM-PMF achieved a more significant performance when it was applied to categorical sparse data conditions, such as data training ratio of 10 : 90, 20 : 80, and 30 : 70, in both ML-1M and ML-10M. CNN-PMF is another document latent representation model that supports matrix factorization work on sparse data. CNN is a subclass of deep learning machine with a specific ability in dimensional reduction features. Compared with another traditional BOW method, CNN showed better performance in various scenario training sets and datasets. CNN has also claimed to reach the best performance in generating rating predictions in recent years. In this experiment, we demonstrated a comparison between LSTM-PMF and CNN-PMF. Surprisingly, LSTM-PMF was superior over CNN-PMF in every section of the training set scenario, including ML-1M and ML-10M. LSTM-PMF achieved 0.71% and 1.4% on average. The competition of LSTM-PMF and CNN-PMF resulted in dimensional reduction and sequential aspect information. Finally, LSTM-PMF performed better in comparison to other competitors due to LSTM's sequential role mechanism; that is, it was more representative in capturing the contextual understanding of the product review documents.

## 4. Conclusion

Sparse data issues caused due to a minimum rating are a major concern in the recommender system. In this research, we proposed a latent factor model using LSTM, word embedding, and PMF. LSTM and word embedding consider word sequential to interpret document understanding to capture the contextual insight of the product review documents. According to our experiment report, our model was superior over previous works. It was believed that the superior performance of LSTM-PMF was due to the impact of the contextual insight representation of the document in supporting the latent factors based on PMF in increasing the effectiveness in generating ratings. Moreover, the involvement of product documents using LSTM and GLOVE also achieved better efficiency in the training process and helped to achieve convergence in an overall training scenario. Contextual insight interpretability can be learnt through bidirectional encoder representation (BERT). Considering the bidirectional model to enhance contextual understanding of the document will possibly improve the matrix factorization performance in predicting the rating matrix. It will become challenging for future research work. PMF is a variant of the matrix factorization method. LSTM-PMF can be expanded by mixing other matrix factorization methods, for example, SVD, SVD++, and nonnegative matrix factorization, that only consider the rating factor. Combining LSTM-PMF with some of the approaches mentioned above can possibly boost the effectiveness of rating prediction with sparse data in large datasets.

## Figures and Tables

**Figure 1:** Collaborative filtering rating matrix.

**Figure 2:** The framework of the LSTM-PMF model including latent factor using PMF and capturing the contextual understanding of the document using LSTM.

**Figure 3:** The common approach of the latent factor model using matrix factorization to produce rating prediction.

**Figure 4:** Basic concept of LSTM work.

**Figure 5:** Capturing contextual insight using GLOVE and LSTM.

**Figure 6:** Hybridization scenario for GLOVE, LSTM, and PMF.

**Figure 7:** Evaluation of LSTM-PMF on ML-1M 10/90.

**Figure 8:** Evaluation of LSTM-PMF on ML-1M 20/80.

**Figure 9:** Evaluation of LSTM-PMF on ML-1M 30/70.

**Figure 10:** Evaluation of LSTM-PMF on ML-1M 40/60.

**Figure 11:** Evaluation of LSTM-PMF on ML-1M 50/50.

**Figure 12:** Evaluation of LSTM-PMF on ML-1M 60/40.

**Figure 13:** Evaluation of LSTM-PMF on ML-1M 70/30.

**Figure 14:** Evaluation of LSTM-PMF on ML-1M 80/20.

**Figure 15:** Evaluation of LSTM-PMF on ML-1M 90/10.

**Figure 16:** Comparison of LSTM-PMF over the state-of-the-art methods ML-1M.

**Figure 17:** Evaluation of LSTM-PMF on ML-10M 10/90.

**Figure 18:** Evaluation of LSTM-PMF on ML-10M 20/80.

**Figure 19:** Evaluation of LSTM-PMF on ML-10M 30/70.

**Figure 20:** Evaluation of LSTM-PMF on ML-10M 40/60.

**Figure 21:** Evaluation of LSTM-PMF on ML-10M 50/50.

**Figure 22:** Evaluation of LSTM-PMF on ML-10M 60/40.

**Figure 23:** Evaluation of LSTM-PMF on ML-10M 70/30.

**Figure 24:** Evaluation of LSTM-PMF on ML-10M 80/20.

**Figure 25:** Evaluation of LSTM-PMF on ML-10M 90/10.

**Figure 26:** Graphical comparison of LSTM-PMF over the state-of-the-art methods on ML-10M.

**Table 1:** Previous state-of-the-art methods.

Method	Description
SVD	A collaborative filtering recommender system based on the latent factor model that is applied by using singular value decomposition (SVD) as the low-rank dimensional factorization, aimed at generating rating prediction [12]
PMF	An advanced version of the SVD model that considers a probabilistic approach to enhance the correspondent users and items. PMF has become a standard rating prediction approach that only involves ratings for collaborative filtering [15]
LDA	An early proposed model that integrates product review document and matrix factorization and aims to interpret the document by exploiting LDA to increase the effectiveness in rating prediction [16]
CTR	A state-of-the-art recommendation model, which combines collaborative filtering (PMF) and topic modeling (LDA) to utilize both ratings and documents [17]
CDL	Another state-of-the-art recommendation model, aimed at enhancing the accuracy of rating prediction by analyzing product documents using a deep learning machine approach based on the autoencoder (AE) that is integrated into the latent factor based on PMF [18]
DCCR	Deep collaborative conjunction recommender (DCCR), a model resulting from multilayer perceptron (MLP) and autoencoder (AE). The autoencoder is responsible for extracting the latent features of an item representation, and the MLP is responsible for detecting the correspondent user and item based on fusion [19]
ConvMF	A collaborative filtering model that involves the traditional matrix factorization model and the document of a product review. Capturing product document understanding involves the convolutional neural network (CNN) with dimensional reduction feature and word embedding [20]. This model is an enhancement of the CDL and CTR models
Att-ConvCF	A version of the collaborative filtering approach, combining matrix factorization and document product review using the attention method in the convolutional process. Matrix factorization is responsible for producing rating prediction [21]
SRCMF	Social review from customer integrated into matrix factorization to achieve effectiveness in generating rating prediction. This approach also requires a product document to be integrated into matrix factorization [22]

**Table 2:** The improvement of latent factors using contextual insight.

Ref.	Method	Latent factor	Rating	Item side document	Bag of words	Deep learning category		
						AE	CNN	LSTM
[15]	PMF	√	√	—	—	—	—	—
[16]	LDA	√	√	√	√	—	—	—
[17]	CTR	√	√	√	√	—	—	—
[18]	CDL	√	√	√	—	√	—	—
[26]	SVD + AE	√	√	√	—	√	—	—
[20]	CNN + PMF	√	√	√	—	—	√	—
	(LSTM + PMF)	√	√	√	—	—	—	√

**Table 3:** Preprocessing the text document.

Method	Step description
Set the maximum words	The product review contains long sentences. However, in this experiment, this section limits the number of words in a sentence to a maximum of 300 words. In movie reviews, most of them consist of less than 300 words. Based on the above considerations, the number of words is limited to a maximum of 300 words. Following the previous works, this scenario is sufficient to generate information on the user's expression representation
Remove stop words	There are many categories of words that can be selected, such as stop words, to achieve the goal. In the case of search engine applications, there are several existing words, concise purpose words, etc.; for example, there are, in, where, also, and on, and, especially in labels like “the on,” “the also,” “there are,” or “in where.” In another method, a search engine erases some of the most famous words, for instance, lexical words, such as “need” in a query that aims to increase achievement
Remove frequently occurring words	This section removes the data corpus for special stop words for documents that occur frequently (more than 0.5). This process is essential to avoid words that appear too often so that they dominate emergence
Remove non-English vocabulary	This section aims to remove all non-English vocabulary words from a catalog document. As an output, the average number of words per document is 97.09 and 92.05 on the MovieLens dataset 1 million (ML-1M) and Amazon instant video (AIV), respectively. In this section, items without a description document in every dataset catalog, and specifically in the Amazon dataset table, are removed. Besides, users without ratings below three are also removed. As an output, every data table demonstrates three datasets with distinct specifications. Even though many users were removed in preprocessing, the Amazon dataset remained quite lacking over the other data
Remove frequently occurring words	This section removes the data corpus for specifically stop words for documents that frequently occur with more than 0.5. This rule is essential to avoid the word from appearing frequently

**Table 4:** Dataset characteristics.

Data category	Number of users	Number of movies	Number of ratings	Sparsity level (%)	Extra information
1M	6.040	3.544	993.482	4.64	Demographic
10M	69.878	10.073	9.945.875	1.41	95.580 #tags
AIV	29.757	15.149	135.188	0.03	Review

**Table 5:** Tools and library.

Number	Tools and library	Specification
1	Processor	Intel Xeon quad core, 2.4 GHz
2	Memory	32 GB
3	GPU	Nvidia Tesla P100 PCI-E 12 GB
4	Tensor flow	Deep learning tools
5	Keras	Deep learning tools
6	Anaconda	Web interface
7	Python	Tool programming
8	Scikit-learn	Evaluation metrics, ML module
9	Pylearn	
10	Surface	RecSys SVD
11	NLTK	NLP module
12	Matplotlib	Data analytics visualization
13	GLOVE	Word vector representation
14	NumPy	Matrix factorization

**Table 6:** Performance comparison of LSTM-PMF with the state-of-the-art methods on ML-1M.

Sparseness level (high-low)	RMSE evaluation result			Comparison result	
	PMF	CNN-PMF	LSTM-PMF	PMF versus LSTM-PMF (%)	CNN-PMF versus LSTM-PMF (%)
10% (90% sparseness level)	1.64697	0.99541	0.9928	**39.00**	**0.26**
20% (80% sparseness level)	1.26577	0.9276	0.93214	**26.70**	**0.48**
30% (70% sparseness level)	1.1118	0.90507	0.89993	**18.59**	**0.56**
40% (60% sparseness level)	1.03992	0.88525	0.88458	**14.87**	**0.08**
50% (50% sparseness level)	0.99064	0.87787	0.87114	**11.38**	**0.76**
60% (40% sparseness level)	0.95897	0.86774	0.86157	**9.50**	**0.71**
70% (30% sparseness level)	0.93369	0.86874	0.85471	**6.95**	**1.61**
80% (20% sparseness level)	0.91134	0.85574	0.84745	**6.10**	**0.96**
90% (10% sparseness level)	0.90452	0.84971	0.84079	**6.06**	**1.04**
∑ (total)				**139**	**6.46**
$\bar{X}$ (average)				**15.4**	**0.71**

**Table 7:** Performance comparison of LSTM-PMF over the state-of-the-art methods on ML-10M.

Sparseness level (high-low)	RMSE evaluation result			Comparison result	
	PMF	CNN-PMF	LSTM-PMF	PMF versus LSTM-PMF (%)	CNN-PMF versus LSTM-PMF (%)
10% (90% sparseness level)	1.27539	0.93629	**0.95506**	**25.10**	−2
20% (80% sparseness level)	1.05233	0.89332	0.89117	**15.30**	**0.24**
30% (70% sparseness level)	0.96513	0.86621	0.85185	**11.70**	**1.65**
40% (60% sparseness level)	0.91827	0.84673	0.82737	**9.89**	**2.28**
50% (50% sparseness level)	0.88834	0.83604	0.81567	**8.18**	**2.43**
60% (40% sparseness level)	0.86673	0.82794	0.80968	**6.58**	**2.20**
70% (30% sparseness level)	0.85071	0.82054	0.80276	**5.63**	**2.16**
80% (20% sparseness level)	0.84049	0.81276	0.79735	**5.13**	**1.89**
90% (10% sparseness level)	0.82796	0.80505	0.7902	**4.56**	**1.84**
*∑* (total)				**92**	**13**
$\bar{X}$ (average)				**10.23**	**1.44**

## Data Availability

Data used to support the findings of this study are included within the article.

## References

[1] Aggarwal C. C. (2016). *Recommender Systems: The Textbook*.

[2] Uribe C. G., Hunt N., Inc N. (2015). The netflix recommender system: algorithms, business value, and innovation. *ACM Transactions on Information Systems*.

[3] Davidson J., Liebald B., Liu J., Nandy P., Van Vleet T. (2010). The YouTube video recommendation system. *ACM Recsys*.

[4] Schafer J. B., Konstan J. A., Riedl J. (2001). *E-commerce Recommendation Applications*.

[5] Bobadilla J., Ortega F., Hernando A., Gutiérrez A. (2013). Recommender systems survey. *Knowledge-Based Systems*.

[6] Beel J., Gipp B., Langer S., Breitinger C. (2016). Research-paper recommender systems: a literature survey. *International Journal on Digital Libraries*.

[7] Zheng L. (2016). *A Survey and Critique of Deep Learning on Recommender Systems*.

[8] Hanafi M., Suryana N., Sammad Bin A., Hasan A. S. H. (2018). An understanding and approach solution for cold start problem associated with recommender system: a literature review. *Journal of Theoretical and Applied Information Technology*.

[9] Hanafi N., Suryana A., Samad Bin A., Hasan B. (2017). Paper survey and example of collaborative filtering implementation in recommender system. *Journal of Theoretical and Applied Information Technology*.

[10] Ricci F., Rokach L., Shapira B. (2015). *Recommender Systems Handbook*.

[11] Harper F. M., Konstan J. A. (2015). The MovieLens datasets: history and context. *ACM Trans. Interact. Intell. Syst*.

[12] Sarwar B. M., Karypis G., Konstan J. a, Riedl J. T. (2000). Application of dimensionality reduction in recommender system - a case study. *Architecture*.

[13] Koren Y. (2010). Collaborative filtering with temporal dynamics. *Communications of the ACM*.

[14] Koren Y., Ave P., Park F. Factorization meets the neighborhood: a multifaceted collaborative filtering model.

[15] Salakhutdinov R., Mnih A. Probabilistic matrix factorization.

[16] Ling G., Lyu M. R., King I. Ratings meet reviews, a combined approach to recommend.

[17] Wang C., Blei D. M. Collaborative topic modeling for recommending scientific articles.

[18] Wang H., Yeung D. (2014). Collaborative deep learning for recommender systems. https://arxiv.org/abs/1409.2944.

[19] Wang Q., Peng B., Shi X., Shang T., Shang M. (2019). DCCR: deep collaborative conjunctive recommender for rating prediction. *IEEE Access*.

[20] Kim D., Park C., Oh J., Lee S., Yu H. (2016). Convolutional matrix factorization for document context-aware recommendation.

[21] Zhang B., Zhang H., Sun X., Feng G., He C. (2019). Integrating an attention mechanism and convolution collaborative filtering for document context-aware rating prediction. *IEEE Access*.

[22] Wang X., Yang X., Guo L., Han Y., Liu F., Gao B. (2019). Exploiting social review-enhanced convolutional matrix factorization for social recommendation. *IEEE Access*.

[23] Kim Y. Convolutional neural networks for sentence classification.

[24] Wang H., Wang N., Yeung D.-Y. Collaborative deep learning for recommender systems.

[25] Pan Y., He F., Yu H. (2020). Learning social representations with deep autoencoder for recommender system. *World Wide Web*.

[26] Wei J., He J., Chen K., Zhou Y., Tang Z. (2017). Collaborative filtering and deep learning based recommendation system for cold start items. *Expert Systems with Applications*.

[27] Koren Y., Bell R., Volinsky C. (2009). Matrix factorization techniques for recommender systems. *IEEE*.

[28] Hochreiter S., Schmidhuber J. (1997). Long short-term memory. *Neural Computation*.

[29] Blei D. M., Edu B. B., Ng A. Y., Edu A. S., Jordan M. I., Edu J. B. (2003). Latent dirichlet allocation. *Journal of Machine Learning Research*.

[30] Pennington J., Socher R., Manning C. Glove: global vectors for word representation.

[31] Idrissi N., Zellou A. (2020). A systematic literature review of sparsity issues in recommender systems. *Social Network Analysis and Mining*.

[32] McAuley J., Leskovec J. Hidden factors and hidden topics.

[33] Stewart I. (2012). Cups and downs. *The College Mathematics Journal*.

[34] McAuley J. (2021). Amazon product data. https://jmcauley.ucsd.edu/data/amazon/.

[35] Burke R. Hybrid recommender systems: survey and experiments.

[36] Çano E., Morisio M. (2017). Hybrid recommender systems: a systematic literature review. *Intelligent Data Analysis*.

